RETRACTED

# Opioid-Free Labor Analgesia: Dexmedetomidine as an Adjuvant Combined with Ropivacaine

**DOI:** 10.1155/2022/2235025

**Published:** 2022-03-29

**Authors:** Wei Gao, Jie Wang, Zhiguo Zhang, Haiying He, Huiwen Li, Ruili Hou, Liping Zhao, Daniel Muthee Gaichu

**Affiliations:** ^1^Department of Anesthesiology, Baotou Obstetrics and Gynecology Hospital, Inner Mongolia (the Third Hospital of Inner Mongolia Baotou Iron and Steel Group), Gaotou 014010, China; ^2^Department of Neonatal Pediatrics, Baotou Obstetrics and Gynecology Hospital, Inner Mongolia (the Third Hospital of Inner Mongolia Baotou Iron and Steel Group), Gaotou 014010, China; ^3^School of Public Health Baotou Medical College, Gaotou 014010, China; ^4^Department of Gynecology and Obstetrics, Baotou Obstetrics and Gynecology Hospital, Inner Mongolia (the Third Hospital of Inner Mongolia Baotou Iron and Steel Group), Gaotou 014010, China; ^5^Chuka University, Chuka 60400, Kenya

## Abstract

**Background:**

Side effects of the use of opioid analgesics during painless delivery are the main factors that affect rapid postpartum recovery. Opioid use can result in dangerous respiratory depression in the patient. Opioids can also disrupt the baby's breathing and heart rate. The nonopioid analgesic dexmedetomidine, a new a2-adrenergic agonist, possesses higher selectivity, greater analgesic effects, and fewer side effects. Moreover, epidural administration of dexmedetomidine also reduces local anesthetic consumption.

**Objective:**

Our study aims to compare the analgesic effects as well as the side effects of ropivacaine with dexmedetomidine against sufentanyl as an epidural labor analgesia.

**Methods:**

This study is a randomized, double-blinded, controlled trial (registration no. ChiCTR2200055360) involving 120 primiparous (a woman who has given birth once), singleton pregnancy women who are greater than 38 weeks into gestation and have requested epidural labor analgesia. The participants were randomized to receive 0.1% ropivacaine with sufentanyl (0.4 *μ*g/ml) or dexmedetomidine (0.4 *μ*g/ml). The primary outcomes included Visual Analogue Score (VAS), duration of first epidural infusions, the requirement of additional PCEA bolus, and adverse reactions during labor analgesia.

**Results:**

Of the 120 subjects who consented, 91 parturient women (women in the condition of labor) had complete data for analysis. Demographics and VAS, as well as maternal and fetal outcomes, were similar between the groups. The duration of first epidural infusions in dexmedetomidine was significantly longer than sufentanyl (median value: 115 vs 68 min, *P* < 0.01); the parturient women who received dexmedetomidine and who required additional PCEA bolus were fewer in comparison to those who received sufentanyl (27.5% vs 49.0%, *P* < 0.05). Furthermore, the incidence of pruritus in the dexmedetomidine group was lower in comparison to the sufentanyl group (0% vs 11.8%, *P* < 0.05).

RETRACTED

**Conclusions:**

Dexmedetomidine, a nonopioid, is superior to the opioid analgesic sufentanyl in providing a prolonged analgesic effect as an epidural during labor. It also reduces local anesthetic consumption and has fewer side effects. The trial is registered with ChiCTR2200055360.

## 1. Introduction

The pain of childbirth is severe and unbearable to most primiparous women, hence effective labor analgesia options are necessary to improve the intrapartum maternal-fetal well-being [1]. A combination of local anesthetic and an opioid is often administered for the management of severe pain to ensure that a minimal dose of each is used. Ropivacaine, combined with low-dose sufentanyl, has been widely and effectively used to provide analgesia for epidural labor [2]. However, opioids can produce side effects themselves, including vomiting, nausea, pruritus, respiratory depression, urinary retention, and reduced variability in the fetal heart rate [3].

Opioid-free anesthesia (OFA) is a multimode anesthesia strategy that combines multiple nonopioid drugs and/or techniques to obtain high-quality anesthesia and has recently gained increasing attention [4]. The impact of OFA has been investigated in the case of transthoracic oesophagectomy in comparison with opioid-based anesthesia technique (OBA) on postoperative analgesia and recovery criteria (hemodynamics, respiratory rate, and hemoglobin oxygen saturation) [5].

As a new agonist of the a2-adrenergic receptor, the nonopioid, dexmedetomidine, is characterized by its high selectivity and greater analgesic effects [6, 7]. Dexmedetomidine-based OFA in cardiac surgery patients is feasible and could be associated with lower postoperative morphine consumption and better postoperative outcomes, reducing local anesthetic consumption, as well as producing fewer side effects [8]. Dexmedetomidine has been shown to protect numerous organs in recent studies (such as the heart, kidney, lung, intestine, liver, and nervous system). This mechanism is thought to primarily relate to the regulation of neuro-transmitters and singling pathways, as well as having antiapoptotic and anti-inflammatory properties [9]. Previous studies have indicated that epidural ropivacaine in combination with dexmedetomidine is an effective method of reducing postoperative pain, prolonging the analgesic effect [10]. The purpose of this study was to carry out a randomized, double-blinded, controlled trial for evaluating the maternal and fetal safety, analgesic effects, and adverse effects of dexmedetomidine in comparison to sufentanyl used as an adjuvant to local anesthetics during epidural labor analgesia.

RETRACTED

## 2. Materials and Methods

This study is a randomized, double-blinded, controlled clinical trial with registration no. ChiCTR2200055360 and is approved by the Inner Mongolia Baotou Maternity Hospital's Ethics Committee. Between January 2021 and August 2021, written informed permission was received from 120 study participants who requested epidural labor analgesia. Parturients were enrolled if they were considered as a physical status I or II (according to the American Society of Anesthesiologists), aged between 20 and 36 years, weighed less than 100 kg, carried a single fetus ≥38 weeks, and experienced cervical dilation ≥3 cm and ≤5 cm. The study exclusion criteria included patients with hypertensive disease, multiple gestations, and history of premature labors and patients with contraindications to epidural analgesia or allergies to opioids/local aesthetics, a history of chronic opioid analgesic use, and VAS ≥4 30 min after epidural labor analgesia.

120 patients were randomized in a balanced manner into two groups via a computer-generated random-number table: the sufentanyl group (Group S, *n* = 60) and the dexmedetomidine group (Group D, *n* = 60). All parturients who met the inclusion criteria were established with venous access and had their vital signs monitored (blood pressure, heart rate, blood oxygen saturation (SpO_2_), and cardiotocography (CTG)) after entering the delivery room. Analgesia was administered in the left lateral decubitus position at the estimated level of the L2 to L3 interspace. The epidural space was identified using a loss-of-resistance approach with an 18-gauge Tuohy needle. An epidural catheter was inserted 3 cm cephaladly into the epidural space. After a negative cerebrospinal fluid and blood aspiration test, a test dose of 3 mL (1% lidocaine) was administered for 5 minutes. As the first epidural infusion dosage, Group S participants received 12 mL 0.4 *µ*g/mL sufentanyl in combination with 0.1% ropivacaine, while Group D participants received 12 mL 0.4 *µ*g/ml dexmedetomidine in combination with 0.1% ropivacaine. These mixed solutions were infused by a patient-controlled-analgesia pump (PCEA) when VAS ≥4. The PCEA pump was set to 8 mL/80 min with an 8 mL rescue bolus (lockout 30 minutes) (Group S: PCEA with ropivacaine (0.1%) + sufentanyl (0.4 *µ*g/mL); Group D: PCEA with 0.1% ropivacaine + 0.4 *µ*g/ml dexmedetomidine). Another anesthetist prepared local anesthetic solutions for epidural labor analgesia. The investigators were blind to these solutions.

RETRACTED

## 3. Outcome Measures and Data Collection

During labor, heart rate, blood pressure, SpO_2_, and cardiotocography (CTG) were continuously monitored and recorded; the parturient's pain level was determined using a 10 cm Visual Analogue Score (VAS: 0 cm = no pain; 10 cm = worst possible pain); the enhanced Bromage score is used to grade the motor block caused by intraspinal anesthesia in parturient women. 0, there is no obstruction to movement; 1, the straight leg cannot be lifted and that the feet and knees cannot be moved; 2, inability to straighten a leg or move the knee, as well as the inability to move the feet; 3, limb movement is completely blocked; additionally, the Ramsay Sedation Scale is used to determine a patient's sedation level: 1, anxiety, irritation, and uneasiness; 2, oriented, calm, and cooperative; 3, responsive only to commands; 4, a brisk reaction to a stimulus; 5, a sluggish reaction to a stimulus; 6, no reaction to a stimulus (T0: prior to the block; T1: 30 min after the block; T2: at the start of the second stage of labor).

The duration of the first epidural infusions, requiring additional PCEA bolus and adverse reactions during analgesia, was observed. The adverse reactions included fever, nausea or vomiting, and pruritus.

Neonatal data including Apgar scores at 1 and 5 minutes, immediate umbilical arterial blood gas analysis (pH, lactic acid), and the Neonatal Behavioral Neurological Assessment (NBNA) on the third day and two weeks after birth were also analyzed. Physicians from our hospital's Department of Children Health examined NBNA scores, which included general condition, muscular tension, action behavior, and primitive reflex. Each parameter received a point value between 0 and 2. All parameters were evaluated before sample collection, given that the consent of family members was obtained.

## 4. Statistical Analysis

SPSS (Windows Version 20.0) was used to conduct statistical analysis. The median, mean, percentage, and standard deviation are all used to depict the data. Comparisons between groups were made using the Mann–Whitney *U* test or independent samples *t*-test. The categorical variables were compared between groups using the Fisher's exact probability test and chi-square detection. The repeated data were analyzed using the analysis of repeated measurements of variance.

## 5. Results

### 5.1. Maternal Characteristics and Neonatal Outcomes

A total of 120 parturients were recruited in this study. Ultimately, 91 parturient women were enrolled (Figure 1), who shared similar bodily characteristics, such as age and weight, as well as similar labor characteristics, such as gestational age. Furthermore, the immediate umbilical arterial blood gas findings (pH, lactic acid), Apgar scores, and NBNA scores between the two groups were also similar (Table 1).

RETRACTED

### 5.2. Quality of Labor Analgesia

There was no significant difference between the VAS and maternal or fetal heart rate between the two groups at T0, T1, and T2 (*P* > 0.05) (Table 2, Figure 2). Furthermore, the requirement of additional PCEA bolus (27.5%) by the parturient women in Group D was less than in Group S (49.0%) (*P* < 0.05, Table 3) (Figure 4).

However, compared with Group S, the duration of the first epidural infusions in Group D (median 115 min, 90–130) was greater than in Group S (median 68 min, 60–80) (*P* < 0.001) (Figure 3).

### 5.3. Maternal Side Effects

The incidence of pruritus in Group D was significantly lower than in Group S (0% vs 11.8%, *P* < 0.05); fever, nausea, or vomiting in Group D (2.5% and 2.5%) was reported lower compared to Group S (7.8% and 5.9%) (Table 3, Figure 4).

## 6. Discussion

Opioid-free anesthesia (OFA) is a new concept of analgesic therapy. OFA is fully in line with the concept of accelerated rehabilitation surgery (ERAS), using multimode anesthesia and pain management to significantly improve patient outcomes and reduce the incidence of postoperative adverse reactions and promote patient recovery [11]. As a result, the optimal labor analgesia not only provides adequate analgesia to parturients but also reduces opioid intake without causing adverse effects, allowing for rapid neonatal or maternal postpartum recovery. Such an analgesic agent has a low risk of motor block, vomiting, nausea, pruritus, bradycardia, and most importantly fetal distress [12].

Sufentanyl, an opioid, has been widely utilized as an adjuvant for epidural labor analgesia in combination with ropivacaine. Opioids are well known to produce side effects themselves, such as nausea, vomiting, pruritus, urinary retention, respiratory depression, and decreased fetal heart rate variability.

As a new a2-adrenergic agonist, dexmedetomidine, a nonopioid, possesses a highly selective, sedative, anxiolytic, sympatholytic, and analgesic effect. Its antinociceptive action is a result of stimulation of a2-adrenoreceptors situated throughout the spinal cord and central nervous system [13]. It has been used as an adjuvant in anesthesia and multimodal analgesia because it can enhance sedation and prolong analgesic effects whilst reducing the risk of adverse reactions opioids can cause [10, 14]. Dexmedetomidine decreases heart rate as its concentration increases in the plasma. This is assumed to be caused by the activation of a2-receptors in vascular smooth muscles, resulting in hypertension and peripheral vasoconstriction. This is presumably caused by the baroceptor reflex [15, 16]. Human studies have shown that a small intravenous bolus of dexmedetomidine decreases blood pressure (0.25–1 *µ*g/kg), whereas larger boluses (1–4 *µ*g/kg) lead to a transient increase in blood pressure and occasionally profound reflex bradycardia [17]. Dexmedetomidine's sedative effect is concentration-dependent; plasma concentrations of 0.2–0.3 *µ*g/mL produce considerable and rousable sedation. Deep sedation is thought to occur at plasma concentrations above 1.9 *µ*g/mL, where a patient is not rousable [15].

RETRACTED

In this work, Group S received sufentanyl and ropivacaine for epidural labor analgesia and Group D received dexmedetomidine 0.4 *µ*g/mL plus 0.1% ropivacaine for epidural labor analgesia.

Compared with Group S, Group D participants did not experience pruritus (0% vs 11.8%) and had fewer complications of nausea and vomiting (2.5% vs 5.9%) in concordance with the study [10]. However, this effect may be related to opioid-free anesthesia rather than the specific antiemetic activity of dexmedetomidine [18].

When comparing the use of sufentanyl, we found that the incidence of fever in dexmedetomidine was lower (7.8% vs 5.9%). Fever during labor analgesia is unknown; it could be caused by heat loss, suppression of the thermoregulatory mechanism of the body, or heat redistribution throughout the body. However, intrathecal dexmedetomidine has the potential to impair the body's thermoregulatory center by impairing the transfer of body temperature signals at the spinal cord level [19].

Patients receiving dexmedetomidine received a longer initial infusion time (115 vs 68) compared to patients administered with sufentanyl. Furthermore, Group D parturient women required fewer additional PCEA boluses (27.5% vs 49%) whist experiencing similar analgesic effects, such as the VAS. In addition, the group's patients and fetuses did not experience significant cardiovascular or sedative side effects, which could be because we used 0.4 *µ*g/mL intrathecal dexmedetomidine, which resulted in a relatively lower plasma concentrations [15, 17, 20].

The immediate umbilical arterial blood gas analysis is an important criterion referenced for the clinical evaluation of fetal acid-base balance. Umbilical artery blood gas analysis and lactic measurements can accurately, objectively, and directly reflect fetal intrauterine oxygenation and stay of ischemia; moreover, this method avoids the disadvantages of using the Apgar scoring system alone. In newborns, the reference range for umbilical cord arterial blood gas is pH 7.10∼7.42, and lactic acid 3.0 ± 1.8. According to relevant clinical study results, the factors affecting neonatal asphyxia levels are directly related to lactic acid changes [21, 22]. The Apgar score, another important criterion of neonatal health, assesses a neonate's physiological reflexes, respiration, muscular tension, and circulation status after delivery. NBNA is a scoring system comprising inspection methods and scoring standards pertaining to 20 neurobehavioral tests in China. It has a total score of 40 points, which comprises 5 segments assessing the ability of newborns to adapt to their external environments as well as external stimuli. Passive and active muscle tone, in addition to original reflex status and general response, are also assessed. A newborn with a score of 37 or higher, within one week of birth, is considered normal [23]. In regards to our study findings, there was no significant difference between the group's immediate umbilical arterial blood pH and lactate. Neither was a difference between the groups' Apgar scores at 1.5 min nor NBNA on the third day and two weeks after birth. This showed that the two methods of anesthesia had little impact on the newborn.

RETRACTED

Therefore, the results of this study show that both sufentanyl (0.4 *µ*g/mL) and dexmedetomidine (0.4 *µ*g/mL) as adjuvants to ropivacaine could provide satisfactory epidural labor analgesia. Moreover, dexmedetomidine is superior to sufentanyl in providing prolonged analgesic effects and also reduces local anesthetic consumption and fewer side effects. It is fully in line with the concept of opioid-free anesthesia (OFA) as a basis for successful fast-track surgery.

It is necessary to mention some limitations of the current study. The most important being the limited number of participants involved. Also, the validity of the results requires the study to be performed at multiple sites. Therefore, the effects of dexmedetomidine on the mother and newborn needs further research using multicenter randomized controlled trials as well as a larger sample size.

## 7. Conclusion

0.4 *µ*g/mL intrathecal dexmedetomidine combined with ropivacaine as an opioid-free epidural labor analgesia therapy can provide satisfactory analgesia effective with lower local anesthetic consumption and fewer side effects. It can also accelerate postpartum recovery during delivery.

## Figures and Tables

**Figure 1:** Participant flow diagram.

**Figure 2:** VAS of two groups at T0, T1, and T2. *P* < 0.05 was considered statistically significant.

**Figure 3:** Duration of the first epidural infusions of the two groups.

**Figure 4:** Maternal side effects and those requiring additional PCEA bolus from the two groups.

RETRACTED

**Table 1:** Maternal characteristics and neonatal outcomes.

	Group S (*n* = 51)	Group D (*n* = 40)	*P* value
Age (years)	27.73 ± 3.13	28.68 ± 2.32	0.113
Body mass index (kg/m^2^)	27.70 ± 3.03	27.81 ± 3.13	0.862
Gestational age (d)	276.70 ± 6.89	276.00 ± 6.27	0.615

*Apgar score*			
1 min	9.57 ± 0.92	9.55 ± 0.96	0.925
5 min	9.96 ± 0.19	9.98 ± 0.15	0.710
Umbilical artery pH	7.29 ± 0.08	7.31 ± 0.05	0.057
Lactic acid (mmol/L)	3.68 ± 1.15	3.81 ± 1.22	0.628

*NBNA score*			
Three days	38.12 ± 1.35	37.70 ± 0.99	0.105
Two weeks	38.96 ± 1.17	38.65 ± 0.89	0.166

Data are reported as mean ± SD or numbers. Group S received sufentanyl 0.4 *µ*g/mL plus 0.1%.

**Table 2:** VAS and maternal or fetal heart rate.

	Group S (*n* = 51)	Group D (*n* = 40)	*P* value
*VAS*			
T0	7.78 ± 1.17	7.38 ± 0.83	0.065
T1	1.06 ± 1.25	0.93 ± 0.79	0.559
T2	2.93 ± 1.01	2.85 ± 0.53	0.688

*Maternal heart rate*			
T0	82.88 ± 9.69	81.43 ± 8.715	0.459
T1	81.24 ± 8.24	79.28 ± 8.32	0.265
T2	83.59 ± 8.54	82.98 ± 6.98	0.714

*Fetal heart rate*			
T0	140.18 ± 6.65	142.58 ± 8.53	0.135
T1	141.57 ± 7.25	142.75 ± 9.35	0.499
T2	143.04 ± 9.61	144.15 ± 9.05	0.576

Date are reported as mean ± SD or numbers.

**Table 3:** Quality of labor analgesia and adverse reactions.

	Group S (*n* = 51)	Group D (*n* = 40)	*P* value
The duration of first epidural infusions (min)	68 (60 to 80)	115 (90 to 130)	<0.01
Requiring additional PCEA bolus, *n* (%)	25 (49.0)	11 (27.5)	0.037
Pruritus, *n* (%)	6 (11.8)	0 (0)	0.033
Nausea or vomiting, *n* (%)	3 (5.9)	1 (2.5)	0.682
Fever, *n* (%)	4 (7.8)	**1 (2.5)**	0.380

Date are reported as median (interquartile range) or *n* (%) of the group. *P* < 0.05 is considered statistically significant.

## Data Availability

The data used to support the findings of this study will be provided upon request to authors.
